The article "Effect of Low-Dose Dexmedetomidine Combined with Lumbosacral Plexus Block Guided by Ultrasound Imaging Based on Image Segmentation Algorithm in Fracture Surgery" was retracted in 2023. Reasons: signs of a paper mill; suspected computer-generated content; unreliable results or conclusions; lack of ethics approval or compliance.

# Effect of Low-Dose Dexmedetomidine Combined with Lumbosacral Plexus Block Guided by Ultrasound Imaging Based on Image Segmentation Algorithm in Fracture Surgery

**DOI:** 10.1155/2022/8063874

**Published:** 2022-05-30

**Authors:** Qiang Ji, Feng Wang, Qiang He, Yanhui Li, Yan Ma

**Affiliations:** ^1^Department of Anesthesiology, Hebei Gucheng Hospital, Hengshui 253800, Hebei, China; ^2^Operation Room, Hebei Gucheng Hospital, Hengshui 253800, Hebei, China; ^3^Department of Pain, Hebei Gucheng Hospital, Hengshui 253800, Hebei, China

## Abstract

The aim of this study was to analyze the application of ultrasound-guided low-dose dexmedetomidine combined with lumbosacral plexus block based on artificial intelligence algorithm in the surgical treatment of proximal femoral fractures. 104 patients with proximal femoral fractures were divided into 52 cases in the experimental group (ultrasound-guided lumbosacral plexus block combined with dexmedetomidine based on local fitting image segmentation algorithm) and 52 cases in the routine group (endotracheal intubation and inhalation combined with general anesthesia). An image segmentation algorithm based on local fitting was constructed to enhance the ultrasound image. It was found that in the routine group, the heart rate (HR), systolic blood pressure (SBP), and diastolic blood pressure (DBP) at the beginning of intravenous injection of dexmedetomidine, during skin incision, and half an hour after skin incision were significantly lower than those at admission (*P* < 0.05). The pressing times of patient-controlled intravenous analgesia (PCIA) in the conventional group (17.05 ± 6.85 times) were significantly higher than that in the experimental group (8.55 ± 4.12 times), and the difference was statistically significant (*P* < 0.05). The visual analogue scale (VAS) scores at 1, 5, 10, and 15 after operation in the routine group were significantly higher than those in the experimental group (*P* < 0.05). The number of dizziness, nausea, and vomiting, venous thrombosis of lower limbs, cardiovascular events, and pulmonary infection in the routine group on the 1st, 2nd, and 3rd days after operation were significantly higher than those in the experimental group (*P* < 0.05). In summary, the ultrasound-guided lumbar plexus-sacral plexus block combined with dexmedetomidine anesthesia based on image segmentation algorithm can effectively maintain the hemodynamic stability of patients, with remarkable analgesic effect and high safety.

## 1. Introduction

The proximal femur includes femoral head, femoral neck, and femoral rotator. Its structure is special. It not only bears the vertical downward pressure from the human body but also bears the shear stress imported into the hip joint during activity, so it is prone to fracture of the femoral neck and the rotator position [1,2]. Proximal femoral fractures are very common in the field of orthopedics and often occur in the elderly. Relevant data show that about 100,000 people in the UK have to undergo surgical treatment for proximal femoral fractures each year. The elderly over 65 years old in the world account for about 14% of the total population, and the hip fractures secondary to osteoporosis are up to 1.6 million each year [3]. In the past, although various active treatment measures, prevention programs, and guidelines have been adopted, the mortality rate of patients with proximal femoral fractures has not been significantly reduced. The controversy and research on the treatment of proximal femoral fractures have also been widely concerned. At present, the commonly used clinical treatment is proximal femoral nail antirotation, which has the advantages of low trauma, less bleeding, high fixation success rate, and less postoperative complications [4, 5]. In the operation, spinal anesthesia or general anesthesia is generally used, but these two methods will increase the risk of operation, such as causing vagus nerve disorder, slow recovery of respiratory function, delayed extubation, and eventually leading to pulmonary infection, deep vein thrombosis, and other complications [6]. Peripheral nerve block is to inject local anesthetics into the vicinity of the peripheral nerve trunk and block the conduction of nerve impulses to make the regional anesthesia within the nerve, which is suitable for the operation limited to a certain nerve trunk and nerve plexus [7, 8].

The article "Effect of Low-Dose Dexmedetomidine Combined with Lumbosacral Plexus Block Guided by Ultrasound Imaging Based on Image Segmentation Algorithm in Fracture Surgery" was retracted in 2023. Reasons: signs of a paper mill; suspected computer-generated content; unreliable results or conclusions; lack of ethics approval or compliance.

With the rapid development of imaging technology, the quality of ultrasound imaging has been continuously improved, and the use of ultrasound to guide local anesthesia has become more and more popular. A large number of traditional local anesthesia technologies have realized visualization with ultrasound [9]. At present, ultrasonic guidance technology is widely applied in peripheral nerve block of the head and neck, maxillofacial region, upper and lower limbs, neck, chest, waist and sacral vertebra, and other related parts, which has a very good effect on clinical anesthesia [10, 11]. Ultrasound-guided local anesthesia is considered to be one of the anesthesia skills that must be mastered, which can effectively improve the success rate of the block, shorten the onset time, reduce complications, and reduce anesthetic toxicity [12]. Image segmentation means that the image is divided into several disjoint regions according to the characteristics of gray, color, spatial texture, and geometric shape, so that these characteristics show consistency or similarity in the same region and show obvious differences in different regions. In other words, in an image, the target is separated from the background. There is no widely applicable image segmentation method, and using machine learning to build an image segmentation model has become a hot topic [13–15]. Considering that the original ultrasonic image will have problems such as noise and artifacts that affect the quality, deep learning technology was used to construct an ultrasonic image segmentation algorithm to assist ultrasonic imaging to guide peripheral nerve block anesthesia, so as to better improve the therapeutic effect of patients with proximal femoral fractures.

The article "Effect of Low-Dose Dexmedetomidine Combined with Lumbosacral Plexus Block Guided by Ultrasound Imaging Based on Image Segmentation Algorithm in Fracture Surgery" was retracted in 2023. Reasons: signs of a paper mill; suspected computer-generated content; unreliable results or conclusions; lack of ethics approval or compliance.

In summary, 104 patients with proximal femoral fractures treated with proximal femoral nail antirotation were selected as the research objects. According to the different anesthesia methods, they were divided into the experimental group (52 cases) and the routine group (52 cases). The experimental group was treated with lumbar plexus-sacral plexus block + dexmedetomidine under ultrasound guidance based on an image segmentation algorithm. The routine group was treated with endotracheal intubation and inhalation combined with general anesthesia. In addition, an image segmentation algorithm based on local fitting was constructed to enhance the ultrasonic image. By comparing the hemodynamics, postoperative recovery index, and visual analogue scale (VAS) score of the two groups, the application value of low-dose dexmedetomidine combined with lumbosacral plexus block guided by ultrasound imaging based on an image segmentation algorithm in proximal femoral nail antirotation was comprehensively evaluated, aiming to provide a reference for the surgical treatment of patients with proximal femoral fracture.

## 2. Materials and Methods

### 2.1. Research Objects

In this study, 104 patients with proximal femoral fractures in the hospital from October 15, 2018, to October 20, 2021, were selected as the research objects. All patients were treated with proximal femoral nail antirotation. There were 45 males and 59 females, aged 45–75 years old, with the course of disease of 3–6 months. According to the different anesthesia methods, they were divided into experimental group (52 cases) and routine group (52 cases). The experimental group was treated with ultrasound-guided lumbar plexus-sacral plexus block + dexmedetomidine based on an image segmentation algorithm, and the routine group was treated with endotracheal intubation and inhalation combined with general anesthesia. All patients voluntarily participated and signed informed consent. This study had been approved by the ethics committee of the hospital.

The article "Effect of Low-Dose Dexmedetomidine Combined with Lumbosacral Plexus Block Guided by Ultrasound Imaging Based on Image Segmentation Algorithm in Fracture Surgery" was retracted in 2023. Reasons: signs of a paper mill; suspected computer-generated content; unreliable results or conclusions; lack of ethics approval or compliance.

Inclusion criteria were as follows: (1) proximal femoral fractures were diagnosed; (2) patients who have not received treatment; (3) it is graded as II-IV by the American Society of Anesthesiologists (ASA); (4) patients voluntary signing of informed consent; (5) patients with complete clinical data.

Exclusion criteria were as follows: (1) patients with peripheral neuropathy; (2) patients with coagulation dysfunction; (3) patients with puncture site infection; (4) patients with mental illness; (5) patients' treatment compliance is poor.

### 2.2. Anesthesia Method

Routine group: (1) first, the upper limb vein channel was established for the patients, and the sodium lactate Ringer's solution was injected intravenously. Moreover, the vital signs such as ECG, body temperature, and pulse oxygen saturation were monitored, and the left radial artery was anesthetized locally with 2% lidocaine. (2) Then, 1.6 mg/kg propofol, 0.5 *μ*g/kg sufentanil, 0.05 mg/kg midazolam, and 0.12 mg/kg vecuronium were injected intravenously. (3) Tracheal intubation was performed, then 3 mg/kg propofol was infused intravenously, 1.5MAC sevoflurane was inhaled, and propofol (200 *μ*g/kg/min) was infused intravenously during the operation.

Experimental group: (1) first, the upper limb vein channel was established for the patients, and the sodium lactate Ringer's solution was injected intravenously. In addition, the vital signs such as ECG, body temperature, and pulse oxygen saturation were monitored, and the left radial artery was anesthetized locally with 2% lidocaine. (2) Patients were placed in the lateral position, intravenous infusion of 1 mg midazolam and 5 *μ*g sufentanil, and an oxygen mask was used. (3) Ultrasonic imaging and nerve stimulator were adopted for positioning. (4) The initial current of the nerve stimulator was 1 mA, the frequency was 3 HZ, the quadriceps femoris was contracted, the current of the instrument continued to decrease until the quadriceps femoris no longer contracted, and 15 mL of 0.32% ropivacaine hydrochloride was infused. (5) Then, the sacral plexus between the ilium and sacrum was located by ultrasound and nerve stimulator, and 15 mL of 0.32% ropivacaine hydrochloride was infused. Finally, 0.3 *μ*g/kg/h dexmedetomidine was intravenously injected.

### 2.3. Image Segmentation Algorithm Based on Local Fitting

In the level set active contour image segmentation, the initial contour is generally set to the level set symbol distance function, but with the increase of iteration times, the symbol distance function will gradually degenerate [16]. In order to ensure that the symbolic distance function always meets |∇*η*|=1, an equation of repeated initialization operation is set.

(1) $$\begin{array}{c} \frac{\partial \eta }{\partial t}=\text{sign}\left(\eta_{0}\right)\left(1-\left|\nabla \eta \right|\right), \end{array}$$

*η*_0_ represents a level set, sign(*η*_0_) is a symbolic function, and ∇ a means gradient operator. When the level set is not smooth, it is difficult to accurately locate the target boundary, resulting in the excessive calculation. Therefore, it is necessary to propose a level set penalty term to replace the symbolic distance function. The penalty term can be expressed as follows:

(2) $$\begin{array}{c} H\left(\eta \right)=\int_{\Omega }\frac{\left(\left|\nabla \eta \right|-1^{2}\right)\text{d}i\text{d}j}{2}. \end{array}$$

By derivation of Equation (2), Equation (3) can be obtained.

(3) $$\begin{array}{c} \frac{\partial \eta }{\partial t}=\Delta \eta -do\left(\frac{\nabla \eta }{\left|\nabla \eta \right|}\right), \end{array}$$

(*do*) represents divergence operator, and Δ represents Laplacian operator. The kernel window function is introduced to obtain some image regions. For any pixel *N*(*i*) in the image, the local energy pan function of the two-dimensional weighted window can be expressed as follows:

(4) $$\begin{array}{c} F_{i}\left(e_{1},e_{2},\eta \right)=\alpha_{1}\int_{\Omega 1}G_{\kappa }\left(j-i\right){\left|N\left(j\right)-e_{1}\left(i\right)\right|}^{2}\text{d}j \end{array}$$

(5) $$\begin{array}{c} e_{1}\left(i\right)=\frac{\left\{G_{\kappa }\times \left[L\left(\eta \left(i\right)\right)*N\left(i\right)\right]\right\}}{G_{\kappa }\times L\left(\eta \left(i\right)\right)}, \end{array}$$

(6) $$\begin{array}{c} e_{2}\left(i\right)=\frac{\left\{G_{\kappa }\times \left[\left(1-L\left(\eta \left(i\right)\right)\right)*N\left(i\right)\right]\right\}}{G_{\kappa }\times \left(1-L\left(\eta \left(i\right)\right)\right)}, \end{array}$$

where *G*_*κ*_ represents the kernel window function, *e*_1_ and *e*_2_ indicate the artificial setting parameters, (*F*_*i*_) means the local energy pan-function, *N*(*j*) represents the gray value of pixels, *e*_1_(*j*) means the local fitting weighting value of pixels *N*(*i*) within the level set, and *e*_2_(*j*) indicates the local fitting weighting value of pixels *N*(*i*) outside the level set. In addition, the kernel window function adopts the Gaussian kernel function, and the equation can be expressed as follows:

(7) $$\begin{array}{c} G_{\kappa }\left(i\right)=\frac{\exp\left(-i^{2}/2\kappa^{2}\right)}{\sqrt{2\pi \kappa }}. \end{array}$$

The length constraint (LCT) of the contour curve is added to the model to keep the characteristic of the symbolic distance function. Then, the local energy pan function can be updated to (8).

(8) $$\begin{array}{c} F_{i}\left(\eta \right)=\int_{\Omega }F_{i}\left(\eta ,e_{1}\left(i\right),e_{2}\left(i\right)\right)\text{d}i+\text{LCT}\left(\eta \right)+\lambda H\left(\eta \right). \end{array}$$

Equation (8) is processed by the variational method to obtain the gradient descent function of the model.

(9) $$\begin{array}{c} \frac{\partial \eta }{\partial t}=-\kappa_{\tau }\left(\eta \right)\left(\alpha_{1}z_{1}-\alpha_{2}z_{2}\right)+\kappa_{\tau }\left(\eta \right)do\left(\frac{\nabla \eta }{\left|\nabla \eta \right|}\right)+\lambda \left(\Delta \eta -do\left(\frac{\nabla \eta }{\left|\nabla \eta \right|}\right)\right),\\ z_{1}=\int_{\Omega }G_{\kappa }\left(j-i\right){\left|N\left(i\right)-e_{1}\left(j\right)\right|}^{2}\text{d}j,\\ z_{2}=\int_{\Omega }G_{\kappa }\left(j-i\right){\left|N\left(i\right)-e_{2}\left(j\right)\right|}^{2}\text{d}j. \end{array}$$

The fitting function of the model changes with the pixels. The local image information is obtained by the kernel window, and the penalty term is added to reduce the computational complexity of the level set.

The article "Effect of Low-Dose Dexmedetomidine Combined with Lumbosacral Plexus Block Guided by Ultrasound Imaging Based on Image Segmentation Algorithm in Fracture Surgery" was retracted in 2023. Reasons: signs of a paper mill; suspected computer-generated content; unreliable results or conclusions; lack of ethics approval or compliance.

### 2.4. Observation Indicators

The basic situation of patients (gender, age, height, weight, ASA grade, course of disease, operation time) was recorded. The heart rate (HR), systolic blood pressure (SBP), and diastolic blood pressure (DBP) of patients are recorded at admission, immediately after intravenous infusion of dexmedetomidine, at the time of skin incision, and half an hour after skin incision. VAS was used to evaluate the pain degree at 1, 5, 10, and 15 hours after the operation. The confusion assessment method Chinese reversion (CAM-CR) was used to evaluate the state of consciousness of patients. The use of patient-controlled intravenous analgesia (PCIA) was recorded. The patients were followed up for a long time after the operation. The adverse reaction time, the first feeding time, the first urination time, the first ambulation time, hospitalization time, and hospitalization expenses were recorded.

### 2.5. Statistical Processing

The data were analyzed by SPSS19.0 statistical software. The measurement data were expressed as mean ± standard deviation ($\bar{x}$ ± *s*), and the count data were expressed as a percentage (%). One-way analysis of variance was used for pairwise comparison. The difference was statistically significant when *P* < 0.05.

## 3. Results

### 3.1. Comparison of Basic Data between the Two Groups of Patients

Figure 1 shows the comparison of the basic data of the two groups of patients. The number of males and females, height, weight, age, operation time, course of the disease, ASA grade, and other information in the experimental group were not significantly different from those in the routine group (*P* > 0.05).

The article "Effect of Low-Dose Dexmedetomidine Combined with Lumbosacral Plexus Block Guided by Ultrasound Imaging Based on Image Segmentation Algorithm in Fracture Surgery" was retracted in 2023. Reasons: signs of a paper mill; suspected computer-generated content; unreliable results or conclusions; lack of ethics approval or compliance.

### 3.2. Ultrasound Image Data of Proximal Femoral Fractures

Figure 2 indicates the ultrasonic image data of proximal femoral fractures. There is an uneven flocculent echo in the intermuscular vein, and there is bone nonunion.

### 3.3. Effect Display of Algorithm Image Segmentation

In order to verify whether the proposed image segmentation algorithm based on local fitting had excellent performance, the level set model (CV) and fuzzy C-means clustering algorithm (FCM) were introduced to compare with the proposed algorithm for image segmentation.  Figure 3(a) shows the original ultrasound image, there are a lot of noise and artifacts, details are not clear, and the overall quality is low.  Figure 3(b) shows the result of image segmentation and reconstruction of the CV model. Compared with the original image, the artifacts and noise were reduced to some extent, and the image quality was improved, but the display of details was still not clear enough.  Figure 3(c) shows the result of image segmentation and reconstruction of the FCM model. The artifacts and noise were greatly reduced, and the details were clearly displayed, but the image color was somewhat distorted.  Figure 3(d) shows the image segmentation and reconstruction results of the proposed algorithm. There was almost no artifact and noise, the details were clearly displayed, the overall quality was significantly improved, and there was no image color distortion.

### 3.4. Comparison of Hemodynamic Changes between Two Groups

Figure 4 shows the comparison of hemodynamic changes between the two groups. Intragroup comparison showed that the HR, SBP, and DBP in the routine group were significantly lower at the time of intravenous infusion of dexmedetomidine, during skin incision, and half an hour after skin incision than those at admission, and the difference was statistically significant (*P* < 0.05). In the experimental group, there was no significant difference in HR, SBP, and DBP at the time of intravenous infusion of dexmedetomidine, during skin incision, and half an hour after skin incision versus at admission (*P* > 0.05). The comparison between groups showed that the HR, SBP, and DBP of the routine group were significantly lower than those of the experimental group at the time of intravenous injection of dexmedetomidine, at the time of skin incision, and half an hour after skin incision, and the difference was statistically significant (*P* < 0.05).

### 3.5. Comparison of Postoperative VAS Scores between the Two Groups

Figure 5 suggests the comparison of postoperative VAS scores between the two groups. The VAS scores at 1, 5, 10, and 15 after operation in the routine group were significantly higher than those in the experimental group, and the difference was statistically significant (*P* < 0.05).

The article "Effect of Low-Dose Dexmedetomidine Combined with Lumbosacral Plexus Block Guided by Ultrasound Imaging Based on Image Segmentation Algorithm in Fracture Surgery" was retracted in 2023. Reasons: signs of a paper mill; suspected computer-generated content; unreliable results or conclusions; lack of ethics approval or compliance.

### 3.6. Comparison of PCIA between the Two Groups

Figure 6 shows the pressing times of PCIA in the two groups. The pressing times of PCIA in the routine group (17.05 ± 6.85 times) were significantly higher than those in the experimental group (8.55 ± 4.12 times), and the difference was statistically significant (*P* < 0.05).

### 3.7. Postoperative CAM-CR Scores of the Two Groups

Figure 7 shows the comparison of postoperative CAM-CR score results between the two groups. It showed that the difference in the CAM-CR score at 1 day before operation between the routine group and the experimental group had no statistical significance (*P* > 0.05); the CAM-CR scores at 1, 2, and 3 days after operation in the routine group were significantly higher than those in the experimental group, and the difference had statistical significance (*P* < 0.05).

### 3.8. Comparison of Postoperative Adverse Events between the Two Groups

Figure 8 shows the comparison of postoperative adverse events between the two groups. The routine group had 7 cases of postoperative dizziness, 5 cases of nausea and vomiting, 2 cases of lower limb venous thrombosis, 2 cases of cardiovascular events, and 2 cases of pulmonary infection; the experimental group had 1 case of postoperative dizziness, 0 case of nausea and vomiting, 0 case of lower limb venous thrombosis, 0 case of cardiovascular events, and 1 case of pulmonary infection. The comparison showed that the number of patients with postoperative dizziness, nausea and vomiting, lower limb venous thrombosis, cardiovascular events, and pulmonary infection in the experimental group was significantly lower than that in the routine group, and the differences had statistical significance (*P* < 0.05).

### 3.9. Comparison of Postoperative Recovery Indicators between the Two Groups

Figure 9 shows the comparison of postoperative recovery indicators between the two groups. The first feeding time, first urination time, first off-bed activity time, hospitalization time, and hospitalization costs in the experimental group were significantly lower than those in the routine group, and the differences had statistical significance (*P* < 0.05).

## 4. Discussion

With the rapid development of society, aging has become a worldwide problem. The number of the elderly with proximal femoral fractures has gradually increased. Looking for effective and low side effects of treatment is a hot topic for scholars [17–20]. Therefore, 104 patients with proximal femoral fractures treated with proximal femoral nail antirotation were divided into 52 cases of the experimental group (ultrasound-guided lumbar plexus-sacral plexus block based on image segmentation algorithm + dexmedetomidine) and 52 cases of routine group (endotracheal intubation and inhalation combined with general anesthesia), and the image segmentation algorithm based on local fitting was constructed to enhance the ultrasound image. Firstly, the image segmentation and reconstruction results of the proposed algorithm, CV model, and FCM model were compared. This is similar to the research results of Okada et al. [21]. The proposed algorithm had the most obvious effect on improving the quality of ultrasonic images, which was superior to the traditional algorithm. Comparison of the basic data between the two groups showed that there was no significant difference in the number of males and females, height, weight, age, operation time, course of disease, ASA grade, and other information between the experimental group and the routine group (*P* < 0.05), which provided the feasibility for subsequent study. In terms of hemodynamics, the HR, SBP, and DBP immediately after intravenous injection of dexmedetomidine, during skin incision, and half an hour after skin incision in the routine group were significantly lower than those at admission (*P* < 0.05), while there was no significant difference at each time period in the experimental group (*P* < 0.05). It revealed that the hemodynamics of the patients in the experimental group were more stable, which was similar to the study by Harding et al. [22], and the reason for analysis may be that ultrasound-guided lumbar plexus-sacral plexus block based on an image segmentation algorithm combined with dexmedetomidine anesthesia could reduce the patient's tension and fear due to long-term fixed position and make the blood circulation more stable [23].

The article "Effect of Low-Dose Dexmedetomidine Combined with Lumbosacral Plexus Block Guided by Ultrasound Imaging Based on Image Segmentation Algorithm in Fracture Surgery" was retracted in 2023. Reasons: signs of a paper mill; suspected computer-generated content; unreliable results or conclusions; lack of ethics approval or compliance.

The transmission of pain requires the ventral nucleus of the primary sensory ganglia, spinal dorsal horn, and dorsal thalamus to reach the cerebral cortex, and nerve block is to allow drugs to act directly on sensory nerves in a part of the body to block the transmission of pain excitability, so that pain signals cannot be transmitted to the center, which in turn reduces pain [24, 25]. It found that the VAS scores at 1, 5, 10, and 15 after surgery in the routine group were significantly higher than those in the experimental group, and the difference was statistically significant (*P* < 0.05). It suggested that the analgesic effect of ultrasound-guided lumbar plexus-sacral plexus block based on image segmentation algorithm combined with dexmedetomidine anesthesia was better than that of conventional endotracheal intubation and inhalation combined with general anesthesia in patients. In terms of state of consciousness, the CAM-CR score, the number of cases of dizziness, nausea and vomiting, lower limb venous thrombosis, cardiovascular events, and pulmonary infection at 1, 2, and 3 days after surgery in the routine group were significantly higher than those in the experimental group, and the differences were statistically significant (*P* < 0.05). It indicated that ultrasound-guided lumbar plexus-sacral plexus block based on the image segmentation algorithm combined with dexmedetomidine anesthesia could effectively reduce the side effects caused by general anesthesia and improve the early postoperative state of consciousness changes of patients. Comparison of postoperative recovery indicators showed that the first feeding time, first urination time, first off-bed activity time, hospital stay, and hospitalization costs in the experimental group were significantly lower than those in the routine group, and the differences had statistical significance (*P* < 0.05). It meant that ultrasound-guided lumbar plexus-sacral plexus block based on image segmentation algorithm combined with dexmedetomidine anesthesia could create conditions for early rehabilitation training of patients and then promote the patients to recover as soon as possible after surgery.

## 5. Conclusion

In this work, 104 patients with proximal femoral fracture treated by proximal femoral antirotation intramedullary nailing were selected as the research subjects. All of them underwent ultrasound scan based on local fitting image segmentation algorithm to explore the application effect of different intraoperative anesthesia methods. Finally, it was found that ultrasound-guided lumbar plexus-sacral plexus block based on an image segmentation algorithm combined with dexmedetomidine anesthesia could effectively maintain the hemodynamic stability of patients undergoing proximal femoral nail antirotation, with significant analgesic effect, creating conditions for early rehabilitation training of patients and promoting the recovery of patients as soon as possible after surgery, with high safety. However, there are still some problems that need to be improved. The constructed image segmentation algorithm based on local fitting only shows the ultrasound image segmentation results and lacks the quantitative data results as a support, and due to the small sample size of patients and rough grouping, there is a lack of statistical analysis of the application effect of single ultrasound-guided lumbar plexus-sacral plexus block combined with dexmedetomidine anesthesia, which will be improved. In conclusion, the results provide a data reference for the selection of clinical treatment options for proximal femoral fracture.

The article "Effect of Low-Dose Dexmedetomidine Combined with Lumbosacral Plexus Block Guided by Ultrasound Imaging Based on Image Segmentation Algorithm in Fracture Surgery" was retracted in 2023. Reasons: signs of a paper mill; suspected computer-generated content; unreliable results or conclusions; lack of ethics approval or compliance.

## Figures and Tables

**Figure 1:** Comparison of basic data between the two groups. (a) The number of males and females; (b) age; (c) height, and weight; (d) ASA grade; (e) operation time and course of the disease.

**Figure 2:** Ultrasonic image data of proximal femoral fractures. Male, 60 years old, chief complaint: pain, swelling, deformity, and mobility limitation in the right thigh caused by trauma for 2 days.

**Figure 3:** Image segmentation effect display of different algorithms. A is the original ultrasonic image; B is the CV model segmentation result; C is the FCM model segmentation result; D is the proposed algorithm segmentation result.

**Figure 4:** Comparison of hemodynamic changes between the two groups. (a) is HR; (b) is SBP; (c) is DBP. 0–3 represents at admission, immediately after intravenous injection of dexmedetomidine, at the time of skin incision, and half an hour after skin incision, respectively. ^*∗*^Statistically significant difference from 0 (*P* < 0.05); #statistically significant difference from the routine group (*P* < 0.05).

**Figure 5:** Comparison of postoperative VAS scores between the two groups. ^*∗*^The difference was statistically significant *P* < 0.05compared with the routine group ().

**Figure 6:** Pressing times of PCIA in the two groups. ^*∗*^Difference was statistically significant compared with the routine group (*P* < 0.05).

**Figure 7:** Comparison of postoperative CAM-CR score results between the two groups. 0–3 represents 1 day before surgery, 1 day after surgery, 2 days after surgery, and 3 days after surgery, respectively. ^*∗*^Statistically significant difference from the routine group (*P* < 0.05).

**Figure 8:** Comparison of postoperative adverse events between the two groups. (a) Dizziness, nausea and vomiting, lower limb venous thrombosis; (b) cardiovascular events, pulmonary infection. ^*∗*^Statistically significant difference from the routine group (*P* < 0.05).

**Figure 9:** Comparison of postoperative recovery indicators between the two groups. (a) Time to first feeding, time to first urination, and time to first ambulation; (b) hospitalization time and hospitalization costs. ^*∗*^Statistically significant difference from the routine group (*P* < 0.05).

## Data Availability

The data used to support the findings of this study are available from the corresponding author upon request.

## References

[1] Sheehan S. E., Shyu J. Y., Weaver M. J., Sodickson A. D. B. (2015). Proximal femoral fractures: what the orthopedic surgeon wants to know. *RadioGraphics*.

The article "Effect of Low-Dose Dexmedetomidine Combined with Lumbosacral Plexus Block Guided by Ultrasound Imaging Based on Image Segmentation Algorithm in Fracture Surgery" was retracted in 2023. Reasons: signs of a paper mill; suspected computer-generated content; unreliable results or conclusions; lack of ethics approval or compliance.

[2] van der Sijp M., van Eijk M., Tong W. H., Niggebrugge A. (2020). Independent factors associated with long-term functional outcomes in patients with a proximal femoral fracture: a systematic review. *Experimental Gerontology*.

[3] Sawaguchi T., Shigemoto K. (2015). [Hip fracture epidemiology, management and liaison service. multidisciplinary approach for the treatment of proximal femoral fractures]. *Clinical Calcium*.

[4] Tittel S., Burkhardt J., Roll C., Kinner B. (2020). Clinical pathways for geriatric patients with proximal femoral fracture improve process and outcome. *Orthopaedics & traumatology, surgery & research: OTSR*.

[5] Gao Z., Lv Y., Zhou F., Ji H. (2018). Risk factors for implant failure after fixation of proximal femoral fractures with fracture of the lateral femoral wall. *Injury*.

[6] Ponzio D. Y., Shahi A., Park A. G., Purtill J. J. (2015). Intraoperative proximal femoral fracture in primary cementless total hip arthroplasty. *The Journal of Arthroplasty*.

[7] Lawson E., Madougou S., Chigblo P., Quenum G., Ouangré A. F. O., Hans-Moevi Akué A. (2017). Ipsilateral proximal and shaft femoral fractures. *Chinese Journal of Traumatology*.

[8] Zhao R., Cai H., Liu Y., Tian H. K. Z. (2017). Risk factors for intraoperative proximal femoral fracture during primary cementless THA. *Orthopedics*.

[9] Ikeda S. (2015). [Hip fracture--epidemiology, management and liaison service. practice of the secondary fracture prevention of the proximal femoral fracture by the osteoporosis liaison service]. *Clinical Calcium*.

[10] Wang Q., Gu X. h., Li X., Wu J., Wang Q. (2019). Management of low‐energy b proximal femoral fractures by proximal femoral nail anti‐rotation. *Orthopaedic Surgery*.

[11] Berger-Groch J., Hartel M. J., Leiderer M. T., Frosch K.-H. (2020 Jun). Diagnostik und Klassifikation proximaler Femur- und Tibiafrakturen beim Erwachsenen. *Radiologe, Der*.

[12] Cooper A. L., Nagree Y., Goudie A., Watson P. R. G. (2019). Ultrasound‐guided femoral nerve blocks are not superior to ultrasound‐guided fascia iliaca blocks for fractured neck of femur. *Emergency Medicine Australasia*.

[13] Rikli D., Goldhahn S., Blauth M., Mehta S. M. A. (2018). Optimizing intraoperative imaging during proximal femoral fracture fixation - a performance improvement program for surgeons. *Injury*.

[14] Graham S. M., Mak J. H., Moazen M., Leonidou A. (2015). Periprosthetic femoral fracture fixation: a biomechanical comparison between proximal locking screws and cables. *Journal of Orthopaedic Science*.

[15] Söylemez M. S., Fidan F., Polat A., Kazdal C., Kurtan A. (2021). Proximal femoral lateral locking plate versus short cephalomedullary nails for treating AO/OTA 31 A3 intertrochanteric femoral fractures: a retrospective clinical study. *Acta Chirurgiae Orthopaedicae et Traumatologiae Cechoslovaca*.

The article "Effect of Low-Dose Dexmedetomidine Combined with Lumbosacral Plexus Block Guided by Ultrasound Imaging Based on Image Segmentation Algorithm in Fracture Surgery" was retracted in 2023. Reasons: signs of a paper mill; suspected computer-generated content; unreliable results or conclusions; lack of ethics approval or compliance.

[16] Wang X., Zhang Y., Du S. (2021). [Reasons of the guide pin eccentricity of helical blade during proximal femoral nail anti-rotation internal fixation for femoral intertrochanteric fractures]. *Zhongguo Xiu Fu Chong Jian Wai Ke Za Zhi*.

[17] Doğan N., Ertürk C., Gülabi D. (2022). Is proximal femoral nailing of unstable intertrochanteric fractures in the lateral decubitus position without a traction table as safe and effective as on a traction table?. *Injury*.

[18] Calderazzi F., Groppi G., Ricotta A., Ceccarelli F. (2014). Does hip osteoarthritis have a protective effect against proximal femoral fractures? a retrospective study. *HIP International*.

[19] Kang L., Liu H., Ding Z., Ding Y. W. J. (2020). Ipsilateral proximal and shaft femoral fractures treated with bridge-link type combined fixation system. *Journal of Orthopaedic Surgery and Research*.

[20] Yang T.-C., Tzeng Y.-H., Wang C.-S., Lin C. (2019). Are proximal screws necessary for osteosynthesis of stable-stem periprosthetic femoral fractures fixed with non-locking plate and cable?. *Injury*.

[21] Okada T., Iwasaki Y., Koyama T., Sugano N. K. Y. (2009). Computer-assisted preoperative planning for reduction of proximal femoral fracture using 3-D-CT data. *IEEE Transactions on Biomedical Engineering*.

[22] Harding J., Chesser T. J. S., Bradley M. (2013). The Bristol hip view: its role in the diagnosis and surgical planning and occult fracture diagnosis for proximal femoral fractures. *The Scientific World Journal*.

[23] Keyak J. H. (2001). Improved prediction of proximal femoral fracture load using nonlinear finite element models. *Medical Engineering & Physics*.

[24] Wu Z., Yi X., Li Y., Mao C. (2020). Decreased radiation exposure using ultrasound-assisted reduction and fixation of femoral shaft fractures in children: a pilot study. *Ultrasound in Medicine and Biology*.

[25] Kellock T. T., Khurana B., Mandell J. C. (2019). Diagnostic performance of ct for occult proximal femoral fractures: a systematic review and meta-analysis. *American Journal of Roentgenology*.

